The article "Immunotherapy Mechanism of Esophageal Squamous Cell Carcinoma with the Effect of STK11/AMPK Signaling Pathway" was retracted in 2024. Reasons: signs of a paper mill; suspected computer-generated content; unreliable results or conclusions; concerns about the data.

# Immunotherapy Mechanism of Esophageal Squamous Cell Carcinoma with the Effect of STK11/AMPK Signaling Pathway

**DOI:** 10.1155/2022/8636527

**Published:** 2022-04-15

**Authors:** Yang Xia, Peng Wang, Yunyao Ye, Sihui Zhang, Guangzhi Sun, Jie Xu, Gaohua Han

**Affiliations:** Department of Oncology, Taizhou People's Hospital, Taizhou, 225300 Jiangsu Province, China

## Abstract

This study was aimed at exploring the mechanism of serine threonine protein kinase 11 (STK11)/Adenosine 5′-monophosphate-activated protein kinase (AMPK) signaling pathway after immunotherapy for esophageal squamous cell carcinoma (ESCC), providing basic information for the clinical treatment of ESCC. In this study, tissue specimens from 100 patients with ESCC who underwent surgical treatment in Taizhou People's Hospital (group A) and 20 patients with recurrent or metastatic ESCC who received second-line immunotherapy (group B) were collected. The real-time fluorescent quantitative polymerase chain reaction (PCR) (RT-qPCR) technology was used to detect the expression levels of STK11, interferon-*γ* (IFN-*γ*), interleukin 6 (IL-6), and vascular endothelial growth factor (VEGF) in the tissues. The immunohistochemical staining was used to detect the positive expression levels (PELs) of STK11 and AMPK*α* in the tissues, and immunofluorescence staining was used to detect the PELs Teff cells (CD3 and CD8), Treg cells (CD4 and FOXP3), and neutrophils (CD68 and CD163). RT-qPCR results showed that the expression levels of STK11 and IFN-*γ* in group A were obviously lower, and those of IL-6 and VEGF were much higher in contrast to group B (*P* < 0.05). The results of immunohistochemical staining showed that the number of STK11- and AMPK*α*-positive staining cells in group A was dramatically less than that in group B (*P* <0.05). The results of immunofluorescence staining revealed that the number of positive staining cells for Teff cells, Treg cells, and neutrophils in group A was also less dramatically than that in group B (*P* <0.05). In summary, immunotherapy can play a therapeutic effect on ESCC by regulating STK11/AMPK pathway and immune cell infiltration.

## 1. Introduction

The chest is the location with a high incidence of malignant tumors. The most common malignant tumors are esophageal cancer, lung cancer, and mediastinal tumors, and esophageal cancer is the most important breast malignant tumor [1]. Clinical data show that esophageal cancer is mainly divided into two types: esophageal squamous cell carcinoma (ESCC) and adenocarcinoma. It is more common in men, and the cause is still unclear [2]. Statistics show that the mortality rate of esophageal cancer in China has ranked fourth in the world, and the incidence of ESCC accounts for more than 90% of all esophageal cancer patients [3]. Since the early symptoms of esophageal cancer are not very obvious, gastroscopy and endoscopic biopsy are commonly used methods for screening for esophageal cancer. Nowadays, the main clinical treatment for esophageal cancer is comprehensive treatment [4]. For resectable esophageal cancer lesions, surgical treatment is mainly adopted [5]. However, surgical resection alone cannot achieve satisfactory treatment results. Data shows that patients have a higher probability of local recurrence and distant metastasis after surgical treatment, and the survival rate in the past 5 years after surgery is only about 30% [6].

With the deepening of tumor immunology research, immunotherapy has become an effective means to reduce the overall mortality of esophageal cancer patients. Immunotherapy shows the advantages of strong specificity and low toxic and side effects. It can play a role in eliminating the spread or metastasis of tumor cells by regulating the specific antitumor immune response ability of the body [7]. At the same time, finding immunotherapy targets for esophageal cancer is of great significance for improving the treatment effect and increasing the survival rate. Recent studies have shown that the mutation and inactivation of serine threonine protein kinase 11 (STK11) are closely related to the occurrence of malignant tumors, especially playing an important role in the pathogenesis and outcome of a variety of adenocarcinomas [8, 9]. Studies have shown that the mutation rate of STK11 in sporadic gastrointestinal tumors is about 10% [10]. STK11 is the upstream kinase of Adenosine 5′-monophosphate-activated protein kinase (AMPK). STK11 can activate the AMPK pathway by phosphorylating AMPK and then negatively regulate the activity of mammalian target of rapamycin (mTOR) [11]. AMPK is widely present in eukaryotic cells. It is a ternary complex composed of three subunits of *α*, *β*, and *γ*, and it participates in the processes of cell growth, proliferation, apoptosis, and cell polarity to regulate the tumor growth [12]. This suggests that STK11 may be able to regulate cell polarity and energy metabolism by activating the AMPK signaling pathway.

This study was aimed at exploring the specific role of STK11/AMPK pathway in immunotherapy for ESCC. In this study, ESCC tissues of patients with ESCC and receiving immunotherapy were collected, and the expression levels of related molecules in the STK11/AMPK signaling pathway in the tissues were detected. In addition, the expression changes of immune cells in the tissues of the two groups of patients were explored. This study was to provide a theoretical basis for the mechanism of STK11/AMPK pathway in ESCC and the search for new targeted therapies for ESCC.

## 2. Materials and Methods

### 2.1. Materials

TRIzol reagent was purchased from Sigma, USA; PrimeScript™ RT reagent Kit with gDNA Eraser (Perfect Real Time), TB Green® Premix Ex Taq™ (Tli RNaseH Plus), and diaminobenzidine (DBA) staining solution were purchased from Takara in Japan; hydrogen peroxide blocking endogenous peroxidase;,STK11 and AMPK*α* immunohistochemical primary antibodies; secondary antibodies; and Teff cells, Treg cells, and neutrophil immunofluorescence staining primary and secondary antibodies were purchased from ThermoFisher, USA.

### 2.2. Methods

#### 2.2.1. Sample Collection

Tissue specimens of 100 patients with ESCC who were surgically treated in Taizhou People's Hospital (group A) and those of 20 patients with recurrent/metastatic ESCC who received second-line immunotherapy (group B) were collected. Inclusion criteria were described as follows. (I) Patients were diagnosed with ESCC at the first diagnosis. (II) Patients had complete follow-up treatment. (III) Patients undergoing surgery had received radiotherapy, chemotherapy, or other antitumor treatment before treatment. (IV) Patients with recurrent/metastatic ESCC were diagnosed as recurrence or metastasis by ultrasound endoscopy after receiving immunotherapy. (V) Patients and their family members had signed the treatment consent forms. (VI) PS score of patient was less than or equal to 2 minutes. Exclusion criteria were defined as follows: (I) patients with other malignant tumors; (II) patients with serious diseases of the heart, kidney, liver, and other major organs; (III) patients with expected survival period shorter than 3 months; and (IV) patients with incomplete clinical data. The basic information of the two groups of patients is shown in Table 1, which showed that there was no difference between the basic data of the patients (*P* > 0.05). After all specimens were washed with phosphate buffer solution (PBS), they were divided into two parts. Some tissues were stored in liquid nitrogen for subsequent detection of the mRNA level of the target gene, and the left tissues were embedded in paraffin and made into paraffin sections with a thickness of 4 *μ*m for subsequent immunohistochemistry and immunofluorescence staining.

#### 2.2.2. RT-qPCR

The tissues were placed in a centrifuge tube, added with an appropriate amount of TRIzol reagent and mixed well, and lysed at room temperature for 5 minutes. After 1/5 volume of chloroform solution was added, they were shaken vigorously and then allowed to stand at room temperature for 5 minutes and then centrifuged at 12,000 rpm at 4°C for 15 minutes. After the supernatant was removed, an equal volume of isopropanol should be added to mix well and allowed to stand on ice for 20 minutes and centrifuged at 4°C at 12,000 rpm for 10 minutes to discard the supernatant. Next, the tissues were added with an appropriate amount of precooled 75% ethanol solution to wash the precipitate and centrifuged at 4°C at 12,000 rpm for 5 minutes, which was repeated 3 times. After the precipitate was dried, it was added with RNase-free ultrapure water to dissolve. The appropriate amount of RNA was removed, and the reverse transcription of complementary deoxyribonucleic acid (cDNA) was performed according to the instructions of the cDNA reverse transcription kit. The quantitative primer sequences of STK11 interferon-*γ* (IFN-*γ*), interleukin 6 (IL-6), and vascular endothelial growth factor (VEGF) and U6 were designed and synthesized by Sangon Biotech in Shanghai. The primer information is shown in Table 2. U6 was undertaken as the internal reference gene, and the relative expression of the target gene was calculated according to the equation 2^-*ΔΔ*CT^.

#### 2.2.3. Immunohistochemical Staining

The prepared tissue paraffin sections were soaked in xylene solution for 10 minutes, and the tissues were dehydrated by soaking in 100%, 95%, 80%, and 70% ethanol solutions for 2 minutes and then rinsed with distilled water for 5 minutes. After the hydrogen peroxide was added to block the endogenous peroxidase, the tissues were incubated at room temperature for 10 minutes in the dark, rinsed with distilled water for 5 minutes, and then performed with the antigen retrieval treatment. Next, after rinsing with PBS for 5 minutes, the tissues were added with serum homologous to the secondary antibody and then placed in a 37°C environment for enclosed treatment for 15 minutes. After adding with the primary antibody dropwise, the tissues were placed in a refrigerator at 4°C overnight and rinsed with PBS for 5 minutes. At this time, the tissues were added with the chelate containing the secondary antibody and labeled with horseradish peroxidase at the end, incubated at 37°C for 40 minutes, and then rinsed again with PBS for 5 minutes. Finally, they were added with DAB staining solution for color development. The staining results were observed under an optical microscope.

If the cell membrane or cell nucleus was brownish yellow, the staining was positive. The pathologist performed a double-blind reading of the slides and randomly counted each section. 10 high-power fields (400x) containing positive cell staining were selected randomly for each section to count the number of positive cells, and the average value was calculated and recorded.

#### 2.2.4. Immunofluorescence Staining

The paraffin sections were deparaffinized as in step 2.2.3, using CD36 and CD163 cells labeled with M2 macrophages for the target protein located in the cytoplasm. After 0.5% Triton X-100 reagent was added, the paraffin sections were performed with permeate treatment at room temperature for 20 minutes, washed with PBS (3 min × 3), added with goat serum, and blocked at room temperature for 30 minutes. Then, it could add diluted primary antibodies (Teff cells: anti-CD3 and CD8 antibodies; Treg cells: anti-CD4 and FOXP3 antibodies; and M2 type macrophages: anti-CD68 and CD163 antibodies), and the sections were placed in a humidified box, which was put in a 4°C refrigerator to incubate overnight in medium. After washing, the sections were added with diluted secondary antibody containing fluorescent label and incubated in a humid box at 37°C for 1 hour. Then, after the phenyl indole (DAPI) reagent was added after washing, the sections were incubated again for 5 minutes in the dark. After washing, the sections were mounted using a quencher containing antifluorescence to observe the staining results under a fluorescence microscope.

### 2.3. Statistical Analysis

All test data were expressed as mean ± standard deviation, and SPSS 22.0 software was used to analyze and process statistical differences. Differences between groups were compared using independent sample *t* test. When *P* < 0.05, the difference showed a significantly statistical difference, while when *P* < 0.01, the difference was extremely statistically significant.

## 3. Results

### 3.1. RT-qPCR Detection Results of STK11, IFN-*γ*, IL-6, and VEGF in ESCC Tissues

The differences in the expression levels of STK11, IFN-*γ*, IL-6, and VEGF mRNA in ESCC tissues of group A and group B were compared. As can be observed from Figure 1, the expression of IFN-*γ* in esophageal squamous cell carcinoma of group A was significantly lower than that of group B, while the expressions of STK11, IL-6, and VEGF were significantly higher than those of group B. The expression of the internal reference gene U6 in the ESCC tissues of group A and group B was almost the same. U6 was undertaken as the internal reference gene to calculate the relative expression level of each target gene and perform statistical analysis. As revealed in Figure 2, compared with group A, the expression level of IFN-*γ* mRNA in ESCC tissue of group B was extremely significantly increased (*P* < 0.01), while the expression levels of STK11, IL-6, and VEGF mRNA were extremely significantly reduced (*P* < 0.01).

### 3.2. Immunohistochemical Staining to Detect the Positive Expression of STK11 and AMPK*α* in ESCC Tissues

The difference between the number of STK11 and AMPK*α*-positive staining cells in the ESCC tissues of group A and group B was compared, and the results are given in Figure 3. The results shown in Figure 3(a) illustrated that the number of AMPK*α*-positive staining cells in group B was significantly more than that in group A, while the number of STK11-positive staining cells was significantly less than that in group A. 10 staining fields were randomly selected to count the positive staining cells, the average was calculated, and the statistical comparisons were performed. As given in Figures 3(b) and 3(c), compared with group A, the average number of AMPK*α*-positive staining cells in ESCC tissue of group B was extremely significantly reduced (*P* < 0.01), while the average number of STK11-positive staining cells was extremely significantly increased (*P* < 0.01).

### 3.3. Immunofluorescence Staining to Detect the Infiltration of Teff Cells, Treg Cells, and Neutrophils in ESCC Tissue

The differences in Teff cells (CD3 and CD8), Treg cells (CD4 and FOXP3), and neutrophil (CD68 and CD163) immunofluorescence staining in ESCC tissues of group A and group B were compared. It can be clearly seen from Figure 4(a) that the numbers of Teff cells (CD3 and CD8), Treg cells (CD4 and FOXP3), and neutrophils (CD68 and CD163) positive immunofluorescence staining (yellow) cells in group B ESCC tissue were greatly more than those in group A. Therefore, 10 staining fields were randomly selected to count the positive staining cells, and the average was calculated and statistically compared. The results in Figures 4(b), 4(c), and 4(d) suggested that compared with group A, the numbers of positive immunofluorescence cells in Teff cells (CD3 and CD8), Treg cells (CD4 and FOXP3), and neutrophils (CD68 and CD163) creased dramatically in group B patients in ESCC tissues (*P* < 0.01).

## 4. Discussion

Esophageal cancer has gradually become one of the malignant tumors with a high mortality rate in China. Most patients are in the middle and advanced stages when they are diagnosed, and the survival rate of middle and advanced patients in the past 2 years is less than 15% [13, 14]. At present, surgical treatment of esophageal cancer has certain limitations, and the metastasis, recurrence, and mortality in the past 5 years are relatively high [15]. The survival rate of radiotherapy for early esophageal cancer can reach 80%, but due to the high degree of malignancy of the disease, problems such as recurrence and metastasis are prone to occur [16]. Therefore, finding effective treatment methods or treatment targets is of great significance for improving the survival rate of patients with esophageal cancer.

In recent years, STK11, as a newly discovered tumor suppressor gene, has received widespread attention. STK11 germline mutation is the main pathogenic gene of Peutz-Jeghers syndrome (PJS), and the incidence of tumors in PJS patients is 10-18 times that of the general population [17, 18]. Studies have shown that STK11 is involved in the occurrence, development, and differentiation of lung cancer and other cancers [19]. It mainly activates threonine at position 172 on the ring by phosphorylation of AMPK*α* subunit and then plays the role of activating the AMPK pathway [20]. It is not known whether the STK11/AMPK pathway can participate in the treatment effect of ESCC. Based on this, this study adopted ESCC patient tissue as a research sample to analyze the expression of related molecules in the STK11/AMPK pathway and the role of immune cells infiltrating tumors after receiving immunotherapy.

IFN-*γ* plays an important role in tumorigenesis and tumor immunity. Its main antitumor activity is manifested in inhibiting tumor cell proliferation, prolonging cell cycle, inhibiting oncogene expression, activating immune cells (macrophages and NK cells, etc.), and inducing tumor necrosis factor expression and other directions [21, 22]. Wang et al. [23] confirmed that the expression level of IFN-*γ* was significantly increased in patients with esophageal cancer. IL-6 is a kind of cytokine with multiple potency, which can activate the tumor regulation-related protein state on the cell surface by forming a complex and then exert the ability to regulate cell proliferation, migration, and invasion [24]. Research by Qiu et al. [25] showed that the level of IL-6 mRNA in esophageal cancer tissues was significantly higher than that in normal tissues. VEGF is a type of cytokine secreted by vascular endothelial cells that promotes cell division. Many studies have shown that the expression level of this gene in tumor tissues is significantly higher than that in normal tissues [26, 27]. And studies have confirmed that VEGF can be used as an independent prognostic factor for esophageal cancer, which is closely related to tumor burden, lymph node metastasis, and recurrence [28]. The results of this study showed that IFN-*γ* levels in ESCC tissue increased after immunotherapy, while the levels of STK11, IL-6, and VEGF decreased (*P* < 0.05). This may be because immunotherapy regulates the collective immunomodulatory activity, enhances the ability of T cells, improves the phagocytic activity of macrophages, promotes the formation of antibodies, and ultimately enhances the immune ability of the body [29]. In addition, this study used immunohistochemistry to detect the positive expression levels of STK11 and AMPK*α* in ESCC tissues. The results showed that the positive expression levels of AMPK*α* in ESCC tissues increased significantly after immunotherapy, while the positive expression levels of STK11 decreased significantly (*P* < 0.05). It shows that immunotherapy can inhibit the process of ESCC by activating the STK11/AMPK signaling pathway.

Studies have shown that immune cell infiltration in tumor tissue is closely related to the prognosis of patients [30]. The results of tumor immunology research show that the occurrence and development of tumors are related to the disorder or loss of the immune system of the body [31]. Teff cells, Treg cells, and neutrophils are all important immune cell subgroups, which play important roles in maintaining the homeostasis of the body's environment and tumor immune surveillance and resisting autoimmune system diseases [32]. Studies have shown that the levels of Treg and other cells in the peripheral blood or tissues of patients with esophageal cancer are significantly higher than those in healthy people [33]. This may be because when tumors appear in the body, tumor cells can release tumor-related antigens, which in turn induces the proliferation and activation of immune cells. The results of this study showed that Teff cells, Treg cells, and neutrophils PEL in ESCC tissues after immunotherapy were obviously higher than those in normal ESCC tissues (*P* < 0.05). Such results suggest that immunotherapy can inhibit tumor cells by enhancing the immune response of the body, so the levels of Teff cells, Treg cells, and neutrophils in the body have increased.

## 5. Conclusion

This study was aimed at exploring the effects of immunotherapy on the STK11/AMPK pathway, tumor-related cytokines, and immune cell levels in ESCC patients. The results showed that immunotherapy can significantly affect the expression level of tumor-related factors, inhibit the activation of STK11/AMPK signaling pathway, and increase the level of immune cells in the body. However, the results of this study still had some limitations. For example, it only explored the effects of immunotherapy on the levels of related factors and immune cells in patients with ESCC, but it could not prove that the STK11/AMPK signaling pathway can directly participate in the immunotherapy effect of ESCC. In future research, it will prepare corresponding animal or cell models to explore the effect of inhibiting or promoting the expression of STK11/AMPK on the effect of immunotherapy for ESCC. In summary, the results of this study could provide a theoretical reference for understanding the mechanism of action of the STK11/AMPK pathway on ESCC.

## Figures and Tables

**Figure 1:** Agarose gel electrophoresis detection image of the target gene. Note: 1, 2, and 3 represented three parallel samples in the same group.

**Figure 2:** Differences in the expression levels of STK11, IFN-*γ*, IL-6, and VEGF mRNA in ESCC tissues between the two groups. Note: Panels (a~d) showed the relative expression level of STK11, IFN-*γ*, IL-6, and VEGF, respectively; ^∗∗^ suggested that there was a very significant difference compared to group A (*P* < 0.01).

**Figure 3:** Immunohistochemical staining results of STK11 and AMPK*α* in ESCC tissues of two groups of patients. Note: Panel (a) showed the microscopic observation of STK11 and AMPK*α* immunohistochemical staining (magnification 400x); panel (b) was the average number of STK11-positive staining cells; panel (c) showed the average number of AMPK*α*-positive staining cells; ^∗∗^ suggested *P* < 0.01 compared with group A.

**Figure 4:** The immunofluorescence staining results of Teff cells, Treg cells, and neutrophils in ESCC tissues of two groups of patients. Note: Panel (a) showed the fluorescence microscopic observation of Teff cells, Treg cells, and neutrophil immunofluorescence staining (magnification 400x); panels (b), (c), and (d) were the average number of positive staining cells of Teff cells, Treg cells, and neutrophils, respectively (different immune cells in the figure were coexpressed as yellow fluorescence). ^∗∗^ suggested that compared with group A, there was a very significant difference (*P* < 0.01).

**Table 1:** Basic information of patients.

Item	Group A (*n* = 100)	Group B (*n* = 20)	Statistical value	*P* value
Age (years old)	57.28 ± 8.36	58.21 ± 7.69	0.211	0.893
Males (%)	87 (87.0)	17 (85.0)	-1.092	1.221
History of smoking (%)	53 (53.0)	14 (70.0)	0.109	0.937
History of drinking (%)	76 (76.0)	15 (75.0)	0.188	0.820
Differentiation (%)			0.779	0.421
Low	4 (4.0)	1 (5.0)		
Medium	94 (94.0)	18 (90.0)		
High	2 (2.0)	1 (5.0)		
Staging (%)			-0.927	0.885
I A	0 (0.0)	0 (0.0)		
I B	9 (9.0)	1 (5.0)		
II A	15 (15.0)	3 (15.0)		
II B	20 (20.0)	4 (20.0)		
III A	33 (33.0)	7 (35.0)		
III B	7 (7.0)	1 (5.0)		
III C	16 (16.0)	4 (20.0)		

**Table 2:** Primer information for quantitative detection of target gene.

Gene name	Primer sequence (5′→3′)	Product size (bp)
STK11	F: GTCTGGCTGTAGCACCCTG R: GCAGCACATCGAAGAGAAACT	173

IFN-*γ*	F: AGCGATTCCAGTATCCTCACT R: CCAGGCTAAGCACTAGAAAGAGT	185

IL-6	F: AACAGAGACGGATGCTTCAAAA R: CCCCAGTAAAGTGGTCAAGGAT	395

VEGF	F: ATGTGTGTCCGTCTACAGATGT R: GGAAGTGTGATTGGCAAAACTGA	160

U6	F: GCCAGCTCCTACATCTCAGC R: AGCCTGACTTGCTAGTGGATTAT	211

## Data Availability

The data used to support the findings of this study are included within the article.
